RETRACTED

# Diagnostic Value of Inflammatory Markers and Cytokines in Neonatal Sepsis

**DOI:** 10.1155/2022/4143101

**Published:** 2022-05-11

**Authors:** Lijie Wu, Jinku Li, Lili Ping, Xiaoli Zhang, Lina Zhai, Yanmin Li, Ruimin Zhang

**Affiliations:** ^1^Neonatal Department, Handan Central Hospital, No. 15 Zhonghua South Street, Handan City, Hebei Province, China; ^2^Infection Management Department, Handan Central Hospital, No. 15 Zhonghua South Street, Handan City, Hebei Province, China

## Abstract

**Objective:**

To explore the diagnosis value of inflammatory markers and cytokines in neonatal sepsis.

**Methods:**

In this retrospective analysis, 90 cases of neonatal sepsis admitted to our hospital from April 2019 to April 2021 were included in the observation group, and 70 healthy neonates who received routine physical examinations in our hospital during the same period were recruited as the control group. Comparison and analysis of inflammatory markers and cytokines levels between the two groups were performed on days 1, 3, and 7 after the onset. Flow cytometry was used to measure the white blood cells (WBCs) and percentage of neutrophils (N%), immunoturbidimetry was used to determine C-reactive protein (CRP), immunochromatographic analysis was used to determine procalcitonin (PCT) in plasma, and the enzyme-linked immunosorbent assay was used to determine interleukin-27 (IL-27), interleukin-6 (IL-6), interleukin-10 (IL-10), and tumor necrosis factor-*α* (TNF-*α*).

**Results:**

Compared with healthy controls, neonatal sepsis resulted in significantly higher levels of WBC, N%, PCT, and CRP on days 1, 3, and 7 after onset. The levels of WBC, N%, and PCT were continuously decreased from day 1 to day 7, while the levels of CRP were increased on day 1 and day 3 but declined on day 7 (*P* < 0.05). Compared with healthy controls, patients with sepsis showed higher levels of IL-27, IL-6, IL-10, and TNF-*α* on days 1, 3, and 7 after the onset. The levels of IL-27, IL-6, and IL-10 were increased on day 1 and day 3 but decreased on day 7, and the levels of TNF-*α* were continuously decreased from day 1 to day 7 (all *P* < 0.05).

**Conclusion:**

Neonatal sepsis was associated with fluctuating levels of WBC, N%, PCT, CRP, IL-27, IL-6, IL-10, and TNF-*α* at different time points of disease. The joint detection of the above indices provides a new pathway for the early diagnosis of neonatal sepsis.

## 1. Introduction

Neonatal sepsis is a critical pediatric disease and refers to a systemic toxic inflammatory response triggered by inflammatory infection or definite pathogenic bacterial infection after the invasion of bacteria in the blood [1, 2]. The disease can be life-threatening without effective treatment measures. Blood culture is currently used as a reliable means for diagnosing this disease [3]. However, it has a low positive rate and is time-consuming, which prevents its effective use in the early diagnosis of sepsis [4]. In recent years, biomarker detection in neonatal sepsis has captured clinical attention. Here, 90 cases of neonatal sepsis were recruited to analyze the value of inflammatory indicators and cytokines in the early diagnosis of neonatal sepsis, to provide a reliable basis for clinical treatment.

RETRACTED

## 2. Materials and Methods

### 2.1. Patients Profiles

In this retrospective analysis, 90 cases of neonatal sepsis admitted to our hospital from April 2019 to April 2021 were included in the observation group, and 70 healthy neonates who received routine physical examinations in our hospital during the same period were recruited as the control group. There were 49 males and 41 females in the observation group, the age ranged from 1 to 15 days, with a mean age of (7.21 ± 2.44) days, and the birth weight was 2342 g to 2605 g, with a mean weight of (2560.14 ± 26.10) *g*. In the control group, there were 38 males and 32 females, the age ranged from 2 to 13 days, with a mean age of (7.34 ± 2.50) days, and the birth weight was 2360 g to 2658 g, with a mean weight of (2541.23 ± 25.98) *g*. There was no significant difference in general data between the two groups, and they were comparable. The research was approved by the Ethics Committee of the Handan Central Hospital, no. HD2970-917.

The criteria for diagnosing a child with sepsis: the patient has signs and symptoms of an inflammatory reaction, an infection with hypothermia (rectal temperature below 35.0°C) or fever (rectal temperature above 38.5°C), signs of tachycardia, changes in consciousness, hypoxemia, hyperlactatemia, or a jumpy pulse. Sepsis with concomitant organ dysfunction is considered severe sepsis.

Inclusion criteria: patients who were diagnosed with sepsis confirmed by clinical symptoms and signs and laboratory examinations results in our hospital; who met the relevant diagnostic criteria in the *Expert Consensus on Diagnosis and Treatment of Neonatal Sepsis* (2019 Edition) [5]; with undersigned informed consent provided by their family members were included.

Exclusion criteria: patients with other liver and kidney dysfunction and cardiovascular diseases; with allergic diseases and mental diseases; and with incomplete clinical data were excluded.

### 2.2. Methods

Comparison and analysis of inflammatory markers and cytokines levels between the two groups were performed on days 1, 3, and 7 after the onset. Flow cytometry was used to measure the white blood cells (WBCs) and percentage of neutrophils (N%) of children in the observation group, immunoturbidimetry was used to measure C-reactive protein (CRP), immunochromatographic analysis was used to determine procalcitonin (PCT) in plasma, and the enzyme-linked immunosorbent assay was used to determine interleukin-27 (IL-27), interleukin-6 (IL-6), interleukin-10 (IL-10), and tumor necrosis factor-*α* (TNF-*α*).

RETRACTED

### 2.3. Treatment

Cefoperazone sodium (Pfizer Pharmaceuticals Co. Ltd., approval no. H21021894) and immunoglobulin (freeze-dried intravenous human immunoglobulin) (Tonglu Biopharmaceutical Co. Ltd., approval no. S19983038) were given. The warm measures should be taken for the children, corresponding oxygen inhalation be given, acid-base balance be corrected, water and electrolyte balance of the children be maintained, and microcirculation be improved. In addition, the patient needed to be given anti-infective therapy, and the child was infused with cefoperazone sodium by intravenous injection at a dose of 50 mg/kg, twice a day, for 3 consecutive days. Additionally, immune globulin treatment was given via intravenous infusion at a dose of 400 mg/(L·kg), once a day, for 3 consecutive days.

For adjuvant treatment with traditional Chinese medicine, it should be given according to the doctor's order, with a small amount and high frequency. For those who had difficulty taking medicine, enema or nasal feeding could be used instead.

The patients were also given 10 mL of Huanglian Jiedu Decoction, three times daily. The medicinal herbs, including 3 g each of Coptidis Rhizoma and Radix Scutellariae, 5 g each of Fructus Gardeniae and Rhei Radix et Rhizoma, 10 g each of Herba Artemisiae Scopariae, and Lonicerae Japonicae Flos, were decocted with water and filtrated to obtain 30 mL of decoction for administration.

### 2.4. Statistical Analysis

All the obtained data were analyzed using the SPSS 22.0 software (IBM, Armonk, NY, USA). The measurement data are expressed as the mean ± standard deviation. An independent sample *t*-test was used for intergroup comparisons, and one-way analysis of variance was used for multitime point comparison, followed by a student's *t*-test. Differences were considered statistically significant at *P* < 0.05.

## 3. Results

### 3.1. WBC, N%, PCT, and CRP

Compared with healthy controls, neonatal sepsis resulted in significantly higher levels of WBC, N%, PCT, and CRP on days 1, 3, and 7 after onset. The levels of WBC, N%, and PCT were continuously decreased from day 1 to day 7, while the levels of CRP were increased on day 1 and day 3 but declined on day 7 (*P* < 0.05) (Table 1).

### 3.2. IL-27, IL-6, IL-10, and TNF-*α*

Compared with healthy controls, patients with sepsis showed higher levels of IL-27, IL-6, IL-10, and TNF-*α* on days 1, 3, and 7 after the onset. The levels of IL-27, IL-6, and IL-10 were increased on day 1 and day 3 but decreased on day 7, and the levels of TNF-*α* were continuously decreased from day 1 to day 7 (all *P* < 0.05) (Table 2).

RETRACTED

## 4. Discussion

Neonatal sepsis induces a systemic inflammatory response and may predispose to neonatal death in severe cases. Anti-infection treatment is frequently used for disease control in clinical practice [6–8]. However, despite the remarkable outcome, anti-infection treatment is associated with drug resistance, which compromises the treatment outcome [9]. Thus, there exists an urgent need to explore appropriate indicators for rapid and accurate diagnosis of neonatal sepsis.

WBC and N% are reliable indicators to determine infection but are vulnerable to multiple factors, thus presenting marked individual variance [10]. In this study, the WBC and N% levels of the observation group on days 1, 3, and 7 after disease onset were higher than those of the control group and continuously decreased from day 1 to day 7, suggesting a comparatively low diagnostic accuracy of WBC and N% in neonatal sepsis. To our knowledge, CRP is a common acute phase reaction protein with increased levels after inflammation or infection, especially after bacterial infection. Its levels reach a peak at 2 days after infections and return to normal after 7 days [11, 12]. Nevertheless, the changes in the CRP level are insensitive to viral infection but to some noninflammatory diseases such as trauma. Therefore, the stand-alone detection of CRP for the diagnosis of neonatal sepsis is unsatisfactory. The results of the present study showed that compared with the control group, the levels of CRP in the observation group were higher on days 1, 3, and 7 after onset. Its levels increased on day 1 and day 3 but declined on day 7. PCT, a polypeptide consisting of 116 amino acid residues, is up-regulated after systemic infection by monocytes in the human body. Toxins produced by bacteria have a strong inhibitory effect on PCT degradation into calcitonin, which results in a high PCT level in the body [12]. Therefore, PCT is mostly used for the diagnosis of bacterial infection and other unknown febrile diseases. The results in this study showed that compared with healthy controls, neonatal sepsis resulted in significantly higher levels of PCT on days 1, 3, and 7 after onset, and the levels of PCT were continuously decreased from day 1 to day 7. It suggested that PCT is highly expressed within 6 h following severe infection, with a long detection window, but the clinical value of PCT alone remains modest.

RETRACTED

As a cytokine, IL-6 is closely related to the growth and differentiation of various cells and regulates immune responses. IL-27 is an important factor in the development of immune and inflammatory responses in the body [13]. After the generation of activated dendritic cells and monocytes, IL-27 directly and rapidly acts on the initial CD4+ T cells, enhancing the cellular immune response and protecting the body from excessive damage, while IL-10 is significantly up-regulated and maintained for a long time. TNF-*α* is involved in the inflammatory response and strongly promotes the synthesis and release of prostaglandins [14]. It facilitates the chemokine effect of cells and exerts an anti-infection effect. In the present study, compared with healthy controls, patients with sepsis showed higher levels of IL-27, IL-6, IL-10, and TNF-*α* on days 1, 3, and 7 after the onset. The levels of IL-27, IL-6, and IL-10 were increased on day 1 and day 3 but decreased on day 7, and the levels of TNF-*α* were continuously decreased from day 1 to day 7. Thus, joint detection of the above indicators could be considered for an accurate early diagnosis of sepsis.

Traditional Chinese medicine was used as adjuvant therapy in this study. On the basis of symptomatic treatment, TCM syndrome differentiation and nursing can effectively treat neonatal sepsis [15]. In traditional Chinese medicine, neonatal sepsis is classified as “fetal fever” and “fetal toxin”, which is mostly caused by fever and toxin invasion of the fetus through the mother, or evil fever and toxin after birth. The evil toxin stagnates in the heart and fights against the qi and blood, with external manifestations of fever and cold, yellow skin, and the evil toxin disturbs the heart and mind, resulting in irritability and excessive crying, or drowsiness. In Huanglian Jiedu Decoction, Coptidis Rhizoma, and Radix Scutellariae are bitter-cold in nature, with clearing heat, eliminating fire, and detoxifying effects, Herba Artemisiae Scopariae and Fructus Gardeniae clear heat and dampness, relieve fire and abate the symptoms of yellow skin, Lonicerae Japonicae Flos clears heat and detoxifies the body, and Rhei Radix et Rhizoma clears heat from the internal organs. The adjuvant therapy of Chinese medicine may reinforce the treatment efficiency of sepsis.

## 5. Conclusion

Neonatal sepsis was associated with fluctuating levels of WBC, N%, PCT, CRP, IL-27, IL-6, IL-10, and TNF-*α* at different time points of disease. The joint detection of the above indices provides a new pathway for the early diagnosis of neonatal sepsis.

## Figures and Tables

**Table 1:** Comparison of WBC, N%, PCT, and CRP levels in two groups of children.

Groups	Timing	WBC (×10^9^/L)	N%	CRP (mg/L)	PCT (*μ*g/L)
Observation group(*n* = 90)	Day 1	14.02 ± 4.05	79.23 ± 5.66	15.35 ± 7.11	7.06 ± 3.33
	Day 3	10.61 ± 2.5^a^	73.09 ± 7.06^a^	23.55 ± 12.10^a^	3.45 ± 1.50^a^
	Day 7	8.36 ± 2.43^ab^	68.05 ± 7.84^ab^	10.15 ± 4.23^ab^	1.48 ± 0.71^ab^

Control group(*n* = 70)		7.41 ± 1.79^abc^	60.51 ± 8.43^abc^	7.51 ± 3.61^abc^	0.80 ± 0.33^abc^
F		20.225	12.557	16.278	18.157
*P* value		<0.001	<0.001	<0.001	<0.001

^a^ *P* < 0.05 in comparison with Day 1; ^b^*P* < 0.05 in comparison with Day 3; ^c^*P* < 0.05 in comparison with Day 7.

RETRACTED

**Table 2:** Comparison of the levels of IL-27, IL-6, IL-10, and TNF-*α* in the two groups of children.

Groups	Timing	IL-27 (pg/L)	IL-6 (pg/L)	IL-10 (pg/L)	TNF-*α* (pg/L)
Observation group (*n* = 90)	Day 1	49.25 ± 11.85	57.02 ± 16.74	34.15 ± 13.60	25.02 ± 4.35
	Day 3	274.56 ± 133.02^a^	266.32 ± 110.74^a^	49.10 ± 14.98^a^	20.41 ± 4.26^a^
	Day 7	23.28 ± 11.52^ab^	60.58 ± 14.89^ab^	16.36 ± 7.43^ab^	15.98 ± 3.87^ab^

Control group (*n* = 70)		17.60 ± 7.23^abc^	48.31 ± 9.86^abc^	12.43 ± 5.02^abc^	13.90 ± 4.11^abc^
F		23.557	19.857	26.557	35.447
*P* value		<0.001	<0.001	<0.001	<0.001

^a^ *P* < 0.05 in comparison with Day 1; ^b^*P* < 0.05 in comparison with Day 3; ^c^*P* < 0.05 in comparison with Day 7.

## Data Availability

No data were used to support this study.

## References

[1] Shen W., Wu Y., Sun W. (2017). Clinical significance of combined detection of IL-8, PCT and CRP in the diagnosis of neonatal sepsis. *Advances in Modern Biomedicine*.

[2] Wu B., Zhang R., Xu H. (2017). Analysis of the etiology and drug resistance of 198 cases of neonatal sepsis. *Chinese Journal of Hospital Infectious Diseases*.

[3] Neonatal Group of Pediatrics Branch of Chinese Medical Association (2019). Expert consensus on diagnosis and treatment of neonatal sepsis (2019 edition). *Chinese Journal of Pediatrics*.

[4] Li Y., Chen Y., Jiang S. (2017). Positive blood culture results and drug resistance analysis of 76 cases of neonatal sepsis. *Journal of Bengbu Medical College*.

[5] Hosokawa Y., Shimizu T., Owari T., Otsuka K., Hayashi Y., Fujimoto K (2017). Clinical evaluation of urosepsis in tane general hospital; clinical utility of measurement of procalcitonin. *Hinyokika Kiyo*.

[6] Pons M. J., Gomes C., Aguilar R. (2017). Immunosuppressive and angiogenic cytokine profile associated with Bartonella bacilliformis infection in post-outbreak and endemic areas of Carrion’s disease in Peru. *PLoS Neglected Tropical Diseases*.

[7] Roberts C. A., Durham L. E., Fleskens V., Evans H. G., Taams L. S (2017). TNF blockade maintains an IL-10+ phenotype in human effector CD4+ and CD8+ T cells. *Frontiers in Immunology*.

RETRACTED

[8] Zhang K., Xie R., Li W. (2019). The application value of inflammatory indicators and cytokine detection in the early diagnosis of neonatal sepsis. *Clinical Blood Transfusion and Testing*.

[9] Yang T., Wang J. (2020). Comparison of pathogenic bacteria, cytokines and immune function of sepsis between term and premature infants. *Chinese Journal of Emergency Resuscitation and Disaster Medicine*.

[10] Li J., Zhou Q., Liu L. (2019). iagnostic value of C-reactive protein, interleukin-6 and procalcitonin in neonatal early-onset sepsis. *China Maternal and Child Health*.

[11] Zhou H., Song W., Tang T. (2019). The evaluation value of serum PCT content in neonatal sepsis on the release of inflammatory factors and organ function damage. *Journal of Hainan Medical College*.

[12] Li J., Zhou Q., Guo J. (2020). A comparative study of maternal and infant inflammatory cytokine levels with early-onset sepsis at different gestational ages. *China Maternal and Child Health*.

[13] Guo J., Gao N., Zhu Y. (2020). Detection and clinical significance of T lymphocyte subsets, PCT, CRP, Lac and inflammatory factors in neonatal sepsis. *Hainan Medicine*.

[14] Wang H., Liu X., Liu Y. (2019). Evaluation of the effect of neutrophil CD64 combined with serum MCP-1, IL-8, and IL-10 levels on the diagnostic efficacy of neonatal sepsis. *Experimental and Laboratory Medicine*.

[15] Chang Su, Fan X., Xia J. (2019). Observation on changes of neonatal coagulation and fibrinolysis system with fungal infectious sepsis and its influence on prognosis. *Chinese Journal of Hospital Infection*.

